The article "Development of a Novel Nomogram Incorporating Red Blood Cell Distribution Width-Albumin Ratio for the Prediction of 30-day Mortality in Acute Pancreatitis Patients" was published in 2022. Journal: Emerg Med Int.

# Development of a Novel Nomogram Incorporating Red Blood Cell Distribution Width-Albumin Ratio for the Prediction of 30-day Mortality in Acute Pancreatitis Patients

**DOI:** 10.1155/2022/1573931

**Published:** 2022-11-28

**Authors:** Li-na Pan, Shen-ao Pan, Bu-huai Lei, Guang-liang Hong, Kun-wei Chen

**Affiliations:** ^1^Department of Anesthesiology, The First Affiliated Hospital of Wenzhou Medical University, Wenzhou 325000, China; ^2^The Second Clinical Medical College, Wenzhou Medical University, Wenzhou 325035, China; ^3^Department of Emergency, The First Affiliated Hospital of Wenzhou Medical University, Wenzhou 325000, China

## Abstract

**Purpose:**

The available nomograms used to predict acute pancreatitis (AP) are not comprehensive. We sought to investigate the effect of red blood cell distribution width (RDW)-albumin ratio (RA) on prognosis of patients with AP and develop a new nomogram to identify AP patients at high risk for mortality.

**Methods:**

We used data from the Medical Information Mart for Intensive Care IV version 2.0 (MIMIC-IV v2.0). A total of 487 patients with acute pancreatitis were included. Patients enrolled in the study were randomly assigned to the training set and validation set at a 7 : 3 ratio. According to the 30-day mortality rate, the data were divided into a survival group and a death group. Multivariate logistic regression was used to establish a prognostic nomogram for predicting the 30-day mortality in AP patients. The area under the receiver operating characteristic curve (AUC), calibration curve, the net reclassification improvement (NRI), the integrated discrimination improvement (IDI), and a decision curve analysis (DCA) are used to verify the overall performance of the model.

**Results:**

Among 487 patients, 54 patients died (11.1%). 338 patients were assigned to the training cohort and 149 were assigned to the validation cohort. The multivariate analysis results showed that RA, age, heart rate, temperature, AST/ALT, BUN, hemoglobin, potassium, and bilirubin were independent risk factors. The prediction performance of the newly established nomogram was better than those of other common scoring systems (including SOFA, OASIS, and APSIII). The nomogram suggests that RA (OR = 1.706, 95% CI: 1.367–2.185) is the most significant laboratory test indicator influencing prognosis.

**Conclusion:**

The new nomogram incorporating RA performed well in predicting AP short-term mortality. A prospective study with a larger sample is needed to validate our findings.

## 1. Introduction

Acute pancreatitis is a complicated gastrointestinal-related disease with considerable morbidity and mortality and a fluctuating course that is frequently difficult to predict in its early stages [1, 2]. In particular cases of severe acute pancreatitis (SAP), pancreatic tissue releases activated trypsin and a large number of inflammatory factors, aggravating the inflammatory necrosis of the pancreas and even involving other organs and tissues, with a mortality rate of up to 20% [3]. Although approximately, 80% of these patients eventually develop either mild or moderate symptoms, one in five patients will develop severe pancreatitis. Therefore, improving the ability to diagnose severe pancreatitis early is essential for lowering the death rate from acute pancreatitis.

There are already a number of prediction models or scoring systems available for doctors to use in assessing the severity of AP in its early stages, but none are ideal. The Ranson score, for instance, requires lactate dehydrogenase (LDH) at admission, which is not routinely evaluated in the emergency department of many hospitals and is frequently missed. Too many parameters are included in the Acute Physiology and Chronic Health Evaluation II (APACHE II) score [4], preventing its broad adoption by doctors. Therefore, a more convenient, rapid, and effective assessment method is still needed.

By quantifying the size of peripheral red blood cells, the red blood cell distribution width (RDW), a common blood test item, can indicate the heterogeneity of red blood cell volume [5]. It is widely employed in the early differential diagnosis of anemia [6]. Recent research has revealed a strong correlation between a high RDW and the prognosis of a variety of serious diseases, including cancer [7], cardiovascular diseases [8], ischemic stroke [9], and acute respiratory distress syndrome (ARDS) [10]. RA is the ratio of RDW to albumin, and a study showed that the predictive value of RA in stroke patients is even greater than that of RDW [11]. However, few studies have been conducted on the ratio of RDW to albumin in inflammatory diseases.

A nomogram is a helpful mathematical tool for forecasting certain endpoints, such as the evolution of disease progression or mortality, depending on a number of critical parameters. Researchers frequently use nomograms to calculate the risk of a clinical event occurrence [12]. A total of 487 patients with acute pancreatitis were selected from the MIMIC-IV database for this retrospective study, which aimed to determine the capacity of RA to predict mortality in patients with acute pancreatitis. Simultaneously, multiple independent risk factors, including RA, were integrated to build a prognostic nomogram to improve the prediction of overall survival in AP patients.

## 2. Methods

### 2.1. Sources of Data

All the data for this study were derived from MIMIC-IV (2.0), a public critical care database developed by MIT. The database collected data on 315,640 inpatients at Beth Israel Deaconess Medical Center (BIDMC) from 2008 to 2019. Laboratory tests, treatment records, demographic information, and so on are all examples of data. The database has been thoroughly de-privatized of all personal information. The researcher has completed an ethical training program and has been granted access to the database by the MIT Institutional Review Board (Certificate number: 43700334).

### 2.2. Case Inclusion Criteria

The data were collected from the database using PostgreSQL tools and SQL structured query language, and patients with acute pancreatitis were identified using the ICD-9 diagnosis code (5770). The following patients were omitted from the study: (1) Patients younger than 18 years of age. (2) Patients' hospital stay was less than 24 hours. (3) Red blood cell distribution width and albumin data were missing. (4) Patients with missing information rate >10%. If the patient was hospitalized more than once, only data from the first hospitalization were evaluated.

### 2.3. Data Collection

The extracted data included demographic information, prognostic scoring systems, vital signs, comorbidities, and laboratory findings within 24 hours. Demographic information includes sex and age. The prognostic scoring systems included Sequential Organ Failure Score Assessment (SOFA), Acute Physiology Score III (APS III), and Oxford Acute Disease Severity Score (OASIS). Vital signs include heart rate, mean blood pressure, breath rate, and temperature. Laboratory findings included red blood cell distribution width (RDW), albumin, red blood cell distribution width-albumin ratio (RA), aspartate aminotransferase-alanine aminotransferase (AST/ALT), blood urea nitrogen (BUN), creatinine, blood glucose, hemoglobin, white blood cell count (WBC), platelets, blood calcium, blood sodium, blood potassium, and total bilirubin. Comorbidities include chronic heart failure (CHF), chronic pulmonary disease, liver disease, malignant cancer, diabetes, and sepsis. The primary outcome of this study was 30-day mortality.

### 2.4. Statistical Analysis

This study included variables with a missing rate of less than 10% to reduce the possibility of information bias. In variables that do not fit a normal distribution, we use the median to fill in the missing values. We use the mean to fill in the missing values in variables that fit a normal distribution. The included cases were then randomly assigned in a 7 : 3 ratio to the training cohort and the validation cohort. Continuous variables with a normal distribution were expressed as mean standard deviation (Mean ± SD), and group comparisons were made using the independent sample *T* test. Continuous variables that did not fit the normal distribution were expressed as medians (quartiles), and group comparisons were made using the Mann–Whitney *U* tests. Categorical variables were written as frequency (%), and the chi-square or Fisher's exact test was used to compare groups.

In the training cohort, we utilized univariate and multivariate logistic regression to identify characteristics associated with 30-day mortality in individuals with acute pancreatitis. Variables with a *P* of value less than 0.1 obtained from univariate regression were included in multivariate regression for further analysis. The backward stepwise regression method was applied to a multivariate logistic regression model to select variables in the training cohort. For continuous variables that comprised all independent risk factors in the final model, we tested for multicollinearity amongst prognostic components using variance inflation factor (VIF), and an arithmetic square root of VIF ≥2 was considered as collinearity.

The independent risk factors in the multivariate logistic model were used to construct a nomogram to predict the 30-day survival rate of patients with acute pancreatitis. The area under the receiver operating characteristic curve (ROC-AUC) was used as the evaluation index of the nomogram. The calibration curve was used to evaluate the consistency between the predicted probabilities and the actual results. If the calibration curve is close to the diagonal, the calibration is considered good.

Additionally, net reclassification improvement (NRI) and integrated discrimination improvement (IDI) were utilized to evaluate this nomogram. NRI and IDI reflect the improved performance of the new model in comparison to the old model. NRI was utilized to compare the accuracy of two models. IDI was utilized to assess the effectiveness of the improvements. NRI and IDI are more sensitive to differences in discrimination between two models than AUC. Using a decision curve analysis (DCA), we evaluated the clinical value of the prediction model. DCA shows the clinical validity of the prognostic model by showing the net benefit of clinical action guided by the prognostic model. In this study, SPSS (22.0) and R (4.0.5) were used for statistical analysis and mapping. *P* < 0.05 was considered statistically significant.

## 3. Results

### 3.1. Baseline Characteristics of Patients

A total of 487 eligible patients were screened for this research, comprising 272 males (55.9%) and 215 females (44.1%), with a 30-day mortality rate of 11.1%. 338 patients were assigned to the training cohort and 149 to the validation cohort, and none of the characteristics were significantly different between the two cohorts. The training cohort consisted of 194 (57.4%) males and 144 (42.6%) females, with a median age of 59 years. The validation cohort consisted of 78 (52.3%) males and 71 (47.7%) females with a median age of 58 years.  Table 1 summarizes the baseline characteristics of patients with acute pancreatitis.

### 3.2. Univariate and Multivariate Logistic Regression Analyses

Using univariate logistic regression analysis, we discovered that age, heart rate, MBP, breath rate, temperature, RA, AST/ALT, BUN, creatinine, hemoglobin, WBC, platelet, potassium, bilirubin, CHF, and sepsis were risk variables for 30-day death in patients with acute pancreatitis. We integrated these variables into multivariate logistic analysis, and the results indicated that age, heart rate, temperature, RA, AST/ALT, BUN, hemoglobin, potassium, and bilirubin remained risk factors for mortality in acute pancreatitis patients. Among them, we discovered that RA was strongly associated with 30-day mortality, with an OR of 1.706, implying that every one-point increase in RA increases the probability of death by 70.6%. The VIF was computed, and none of the variables listed above had an arithmetic square root of VIF greater than 2, suggesting that multicollinearity was not present in the model.  Table 2 summarizes the results of univariate and multivariate logistic regression analyses.

### 3.3. ROC Curve Analysis of RA, RDW, Albumin, and Three Scoring Systems

ROC curve analysis of RA, albumin, and RDW showed that the AUC value of RA was 0.771(95% CI: 0.69–0.852) (Figure 1(a)), which was significantly higher than that of RDW (0.704, 95% CI: 0.621–0.786) and albumin (0.714, 95% CI: 0.628–0.8) (Figure 1(a)). Compared with the three scoring systems, the AUC value of RA was higher than that of OASIS (0.746, 95% CI: 0.672–0.819) (Figure 1(b)), but lower than that of SOFA (0.79, 95% CI: 0.716–0.863) and APS III (0.837, 95% CI: 0.777–0.896) (Figure 1(b)).

### 3.4. Prognostic Nomogram for 30-Day Mortality and the Nomogram's Performance

We establish a nomogram prediction model based on the results of a multiple logistic regression model.  Figure 2 depicts the nomogram containing all the independent risk factors. The nomogram suggests that RA (OR = 1.706, 95%CI: 1.367–2.185) is the most significant indicator, along with AST/ALT, age, temperature, BUN, bilirubin, heart rate, potassium, and hemoglobin. Based on the findings of nomogram analysis, the area under the receiver operating characteristic curve (AUC) of the training model for predicting the probability of death within 30 days of acute pancreatitis was 0.891, with a 95% confidence interval of 0.846–0.936 (Figure 3(a)). Compared with SOFA, OASIS, and APS III, the AUC value of the training cohort was significantly improved.  Table 3 summarizes the results of the received operating characteristics curve of the nomogram.

The bootstrap method was used to generate the internal calibration curve, and the calibration curve nearly matched the reference curve, showing that the nomogram's capacity for differentiation and prediction was excellent (Figure 4(a)). We put the verification cohort's information into the nomogram for verification. Results indicated that the AUC for predicting the risk of death was 0.898, with a 95% confidence interval of 0.814–0.982 (Figure 3(b)). The calibration curve for the validation cohort stayed close to the standard curve (Figure 4(b)), which shows that the nomogram is good at making predictions.

After comparing the nomogram with SOFA, OASIS, and APS III, the NRI of the training cohort was 0.35, 0.407, and 0.25, respectively. The NRI of the validation cohort was 0.473, 0.515, and 0.372, respectively. In addition, the IDI of the training cohort was 0.199, 0.249, and 0.159, respectively. The IDI of the validation cohort was 0.355, 0.382, and 0.37, respectively.  Table 3 summarizes the NRI and IDI of the training and validation cohorts. We discovered that both NRI and IDI were positive, indicating that the nomogram had a greater capacity for discrimination than the other three scoring systems. In the DCA curve of Figure 5, when the threshold probability is between 0.4 and 0.8, we find that the DCA curve of the nomogram is higher than that of the three scoring systems. This indicates that clinical interventions guided by nomograms could achieve greater net benefits.

## 4. Discussion

The essence of acute pancreatitis is autodigestion of the pancreatic parenchyma, which means that there is a local inflammatory response but also a systemic inflammatory damage, which can be secondary to serious bacterial infection and multiple organ damage [13]. The severity can range from mild self-limited disease to severe acute necrotizing pancreatitis, which is characterized by systemic complications and multiple organ failure [14]. Simultaneously, individuals with acute pancreatitis frequently advance rapidly, making early misdiagnosis common. Thus, early, accurate, and prompt assessment is critical for patients with acute pancreatitis, since it is the key to reducing mortality. Currently, there is still a dearth of efficient clinical markers for swiftly and sensitively assessing the severity of acute pancreatitis. Even while physical examination, imaging features, blood laboratory testing, and scoring systems such as the Bedside Index for Severity in the Acute Pancreatitis (BISAP) score are currently popular ways to differentiate the severity of acute pancreatitis [15]; these methods have their own set of shortcomings. For instance, abdominal pain is not typical in patients; premature CT examination often cannot confirm the diagnosis and may even lead to a misdiagnosis. Serum amylase and serum calcium have low specificity and are frequently inconsistent with the true severity of the patient's condition. The scoring system is still not sufficiently standardized, which restricts its clinical utility to some extent. Therefore, RA, as a straightforward and easily obtainable static indicator, is an excellent supplement to existing evaluation approaches.

In recent years, a number of diagnostic and prognostic markers, both alone and in combination, have been tested on individuals diagnosed with AP [16–18]. After elevated RDW was established as a predictor of poor outcomes in chronic heart failure in 2007, multiple studies have shown that it is significantly related to short-term mortality outcomes in a range of inflammatory disorders [19, 20]. Additionally, Jin [21] and Zhang's [22] studies demonstrated a strong correlation between RDW and acute pancreatitis mortality. Admittedly, RA's outstanding predictive value is in part due to RDW's excellent forecasting ability. However, whether RA is a more accurate predictor of short-term mortality in acute pancreatitis than RDW remains unknown. As a result, we compared the AUC values of RA, RDW, and albumin in this study and were pleasantly surprised to discover that RA had a significantly better predictive performance than RDW and albumin, indicating that RA is a more optimized predictor than RDW, which may be inextricably linked to albumin's critical protective role in a variety of inflammatory diseases [23, 24]. This result is also similar to that of Zhao's study [11]. Simultaneously, univariate analysis revealed that a decrease in albumin was substantially linked with mortality in this study (Table 1), implying that serum albumin may possibly have a protective effect in patients with pancreatitis. However, the mechanisms underlying the association between RDW and mortality from inflammatory diseases remain unclear. It has been shown in one study that there is a strong, positive, and independent correlation between RDW and traditional inflammatory biomarkers. This may be because inflammation reduces red blood cell survival, resulting in differences in red blood cell volumes and an increase in size heterogeneity among red blood cells [25]. Additional evidence suggests that oxidative stress enhances cellular heterogeneity by affecting erythropoiesis and reducing the half-life of red blood cells in circulation, ultimately resulting in elevated RDW levels [26].

However, it remains challenging to reliably estimate the prognosis of a disease based on a single laboratory marker. Increasing the number of indicators used in a diagnostic procedure can improve either its sensitivity or its specificity, and a nomogram is a visual graph of the findings of a multivariate regression analysis [27]. Because the complicated regression equation is converted into a visual graph by the nomogram, the findings of the regression analysis model are made easier to comprehend, are more intuitive, and are simpler to evaluate for the patient. These are advantages of the nomogram. Therefore, nomograms are accepted by a significant number of researchers involved in clinical medical studies and they are widely applied as a visual statistical model for the purpose of determining the prognosis and risk of disease [28, 29].

In this work, we established a nomogram for the early prediction of death in AP patients based on a large population gathered from a critical disease database. The variables included in the nomogram were RA, age, heart rate, temperature, AST/ALT, BUN, hemoglobin, potassium, and bilirubin. In addition, the clinical indicators and laboratory test data included in this nomogram can be easily obtained. The model was validated, and its predictive performance was comparable to that of current scoring systems.

The roles of BUN and creatinine in predicting the prognosis of AP are still debatable. Both renal damage induced by inflammation and renal hypoperfusion produced by hypovolemia can elevate BUN and creatinine levels. Yang et al. [30] revealed that the predictive value of creatinine was much higher than that of BUN in predicting the short-term mortality of severe acute pancreatitis; however, our results demonstrated that the predictive value of BUN was even higher, which is consistent with Jiang's findings [31]. The relatively plausible explanation for the early increase in BUN is insufficient resuscitation resulting in prerenal azotemia [32]. Multiple prior studies have indicated that high bilirubin is a substantial risk factor for early mortality in AP [33, 34]. When AP develops, bile ducts are clogged, bile cannot be excreted, and bilirubin is retained in liver cells, disrupting the normal metabolism of liver cells and reducing liver function [35]. In our study, in addition to the bilirubin level, we also found that the AST/ALT ratio was an independent risk factor. AST and ALT are typically used to signal liver damage, and alcohol consumption can lead to the development of alcoholic cirrhosis and pancreatitis. Studies have shown that the AST/ALT ratio is closely related to the degree of cirrhosis [36]. Therefore, the elevated AST/ALT ratio in a high number of AP patients may be due to excessive alcohol use. In addition to the abovementioned independent risk variables, blood potassium and heart rate were also incorporated into the prediction model, and an increase in these two indicators suggests that the patient may have had severe internal environment abnormalities, metabolic acidosis, or even shock.

Our study has several strengths. First, we found that RA is a significant independent risk factor that was absent from earlier AP models. Second, we constructed a nomogram with readily accessible parameters. This nomogram presents the probability of AP short-term mortality outcomes and allows practitioners to analyze patient outcomes. The performance of our model is far superior to that of traditional disease severity scores.

However, it is vital to point out some of the study's shortcomings, which are as follows: We should note that because this was a retrospective observational study, there is still the possibility of selection bias and confusion bias in our findings. In regard to the second issue, this study's conclusions are not supported by multicenter clinical data, which raises questions about the validity of these findings. Ideally, we should perform additional multicenter research in the future using a large number of study sites.

## 5. Conclusion

Our study reveal the predictive values of RA in patients with AP. Concurrently, the new nomogram demonstrated good performance in predicting short-term mortality in AP by constructing a nomogram employing RA and a number of other easily accessible clinical parameter relevant to AP prognosis. However, additional confirmation of the present findings requires the conduct of larger prospective investigations with a greater duration of follow-up.

## Figures and Tables

**Figure 1:** ROC curves. (a) ROC curves for the RA, RDW, and albumin. (b) ROC curves for the RA, SOFA, OASIS, and APS III. In both figures, RA had higher AUC values than RDW and albumin. The AUC value of RA is lower than SOFA and APS III but higher than OASIS. ROC, receiver operating characteristic; RA, red blood cell distribution width-albumin ratio; SOFA, sequential organ failure assessment; OASIS, Oxford acute disease severity score; APS III, acute physiology score III.

**Figure 2:** Nomogram predicting 30-day mortality in patients with acute pancreatitis. To use a nomogram, draw a vertical line from each variable up to the point. The resulting value is the patient's score on that variable (i.e., “RA = 8” = 50 points). The scores for each variable were then summarized to obtain a total score corresponding to the 30-day probability of death predicted at the bottom of the nomogram. We then plotted a vertical line from the axis of the total point down to the 30-day survival probability, thus obtaining the 30-day survival probability for this patient. RA, red blood cell distribution width-albumin ratio; BUN, blood urea nitrogen.

**Figure 3:** ROC curves for the nomogram, SOFA, OASIS, and APS III in the training cohort (a) and validation cohort (b). The nomogram includes RA, age, temperature, bun, AST/ALT, hemoglobin, bilirubin, potassium, and heart rate. In both groups, the nomogram had higher AUC values than SOFA, OASIS, and APS III.

**Figure 4:** Calibration plots of the nomogram in the training cohort (a) and validation cohort (b). In both groups, although the apparent and corrected curves deviated slightly from the reference line, they also showed good agreement between observation and prediction.

**Figure 5:** The decision curve analysis curves of medical intervention in patients with the nomogram, SOFA, OASIS, and APS III in the training cohort (a) and validation cohort (b). In both groups, the nomogram had superior standardized net benefit over SOFA, OASIS, and APS III.

**Table 1:** Baseline characteristics of patients with acute pancreatitis.

Variables	All (*n* = 487)	Training cohort (*n* = 338)	Validation cohort (*n* = 149)	*P* Value
*Demographics*				
Age (year)	58.95 (47.16 ∼ 72.35)	59.48 (47.79 ∼ 73.86)	58.2 (45.5 ∼ 70.71)	0.199
Gender (*n*, %)				0.301
Female	215 (44.1%)	144 (42.6%)	71 (47.7%)	
Male	272 (55.9%)	194 (57.4%)	78 (52.3%)	
*Prognostic scoring system*				
APS III	53 (37 ∼ 81)	52 (37 ∼ 82)	53 (37 ∼ 77)	0.974
SOFA	5 (3 ∼ 10)	5 (3 ∼ 10)	6 (2 ∼ 9)	0.773
OASIS	34 (27 ∼ 42)	34 (27 ∼ 42)	33 (27 ∼ 41)	0.462
*Vital signs*				
Heart rate (beats/min)	114 (98 ∼ 130)	114 (98 ∼ 130)	114 (99 ∼ 130)	0.782
MBP (mmHg)	106 (93 ∼ 119)	105 (93 ∼ 119)	106 (94 ∼ 117)	0.865
Breath rate (breath/min)	28 (24 ∼ 33)	29 (24 ∼ 34)	28 (24 ∼ 32)	0.348
T (°C)	37.5 (37 ∼ 38.17)	37.56 (37.06 ∼ 38.11)	37.39 (36.94 ∼ 38.17)	0.308
*Laboratory findings*				
RDW (%)	14.8 (13.8 ∼ 16.1)	14.8 (13.8 ∼ 16.2)	14.8 (13.9 ∼ 16.1)	0.908
Albumin (g/dL)	3 (2.4 ∼ 3.5)	3 (2.4 ∼ 3.5)	3 (2.45 ∼ 3.4)	0.887
RA	5.07 (4.22 ∼ 6.25)	5.05 (4.14 ∼ 6.3)	5.11 (4.34 ∼ 6.15)	0.971
AST/ALT	1.42 (1 ∼ 2.13)	1.4 (0.97 ∼ 2.1)	1.46 (1.02 ∼ 2.21)	0.273
BUN (mg/dL)	24 (14 ∼ 42)	25 (14 ∼ 42)	22 (12 ∼ 41)	0.228
Creatinine (mg/dL)	1.1 (0.8 ∼ 2.2)	1.1 (0.8 ∼ 2.1)	1.1 (0.8 ∼ 2.45)	0.855
Glucose (mg/dL)	153 (114 ∼ 215)	153 (115 ∼ 217)	151 (111 ∼ 215)	0.416
Hemoglobin (g/dL)	10.4 ± 2.05	10.48 ± 2.13	10.45 ± 1.85	0.874
WBC (10^9^/L)	13.5 (9.4 ∼ 19.6)	13.45 (9.48 ∼ 19.53)	13.7 (8.75 ∼ 19.7)	0.676
Platelet (10^9^/L)	171 (111 ∼ 250)	174 (111.75 ∼ 259.25)	162 (108 ∼ 233)	0.503
Calcium (mmol/L)	7.7 (7.1 ∼ 8.3)	7.7 (7.1 ∼ 8.3)	7.7 (6.8 ∼ 8.28)	0.82
Sodium (mmol/L)	137 (134 ∼ 140)	137 (134 ∼ 140)	138 (134 ∼ 140)	0.338
Potassium (mmol/L)	4.3 (3.9 ∼ 4.8)	4.3 (3.9 ∼ 4.8)	4.3 (3.9 ∼ 4.85)	0.894
Bilirubin (mg/dL)	1.2 (0.6 ∼ 3)	1.2 (0.6 ∼ 3.2)	1.1 (0.6 ∼ 2.45)	0.784
*Comorbidities*				
CHF (*n*, %)	87 (17.9%)	59 (17.5%)	28 (18.8%)	0.723
Chronic pulmonary disease (*n*, %)	114 (23.4%)	85 (25.1%)	29 (19.5%)	0.172
Liver disease (*n*, %)	154 (31.6%)	109 (32.2%)	45 (30.2%)	0.654
Malignant cancer (*n*, %)	40 (8.2%)	27 (8%)	13 (8.7%)	0.785
Diabetes (*n*, %)	148 (30.4%)	97 (28.7%)	51 (34.2%)	0.221
Sepsis (*n*, %)	324 (66.5%)	229 (67.8%)	95 (63.8%)	0.39

OASIS: Oxford acute severity of illness score; SOFA: Sequential organ failure assessment; APS III: Acute physiology score III; BUN: Blood urea nitrogen; WBC: White blood cell; RDW: Red blood cell distribution width; RA: Red blood cell distribution width-albumin ratio; CHF: Chronic heart failure.

**Table 2:** Univariate and multivariate logistic regression analysis in patients with acute pancreatitis.

	*Univariate analysis*			*Multivariate analysis*		
	OR (95% CI)	*B*	*P* Value	OR (95% CI)	*B*	*P* Value
Demographics						
Age (year)	1.038(1.016∼1.06)	0.037	0.001	1.061(1.03∼1.097)	0.06	<0.001
Gender (n, %)	0.885(0.452∼1.735)	−0.122	0.723			

Vital signs						
Heart Rate (beats/min)	1.011(0.998∼1.024)	0.011	0.093	1.019(1.002∼1.037)	0.019	0.03
MBP (mmHg)	0.981(0.962∼1.0002)	−0.019	0.052			
Breath rate (breath/min)	1.054(1.009∼1.101)	0.053	0.018			
T (℃)	0.519(0.318∼0.848)	−0.655	0.009	0.574(0.293∼1.047)	−0.555	0.086

Laboratory findings						
RA	1.688(1.407∼2.024)	0.523	<0.001	1.706(1.367∼2.185)	0.534	<0.001
AST/ALT	1.363(1.095∼1.696)	0.31	0.006	1.558(1.186∼2.092)	0.443	0.001
BUN (mg/dL)	1.023(1.013∼1.034)	0.023	<0.001	1.018(1.005∼1.032)	0.018	0.007
Creatinine (mg/dL)	1.2(1.059∼1.359)	0.182	0.004			
Glucose (mg/dL)	1.0001(0.998∼1.002)	0.0001	0.906			
Hemoglobin (g/dL)	0.848(0.722∼0.996)	−0.165	0.044	1.183(0.951∼1.478)	0.168	0.134
WBC (109 /L)	1.024(0.997∼1.052)	0.024	0.084			
Platelet (109 /L)	0.997(0.994∼1.0002)	−0.003	0.07			
Calcium (mmol/L)	0.925(0.675∼1.267)	−0.078	0.626			
Sodium (mmol/L)	0.968(0.915∼1.025)	−0.032	0.267			
Potassium (mmol/L)	1.478(1.103∼1.981)	0.391	0.009	1.386(0.93∼2.023)	0.326	0.094
Bilirubin (mg/dL)	1.085(1.027∼1.146)	0.082	0.003	1.099(1.017∼1.19)	0.095	0.016

Comorbidities						
CHF (n, %)	0.35(0.104∼1.177)	−1.049	0.09			
Chronic pulmonary disease (n, %)	0.718(0.317∼1.624)	−0.332	0.426			
Malignant cancer (n, %)	0.268(0.035∼2.033)	−1.316	0.203			
Liver disease (n, %)	1.151(0.575∼2.303)	0.14	0.692			
Diabetes (n, %)	1.58(0.794∼3.147)	0.458	0.193			
Sepsis (n, %)	2.453(1.049∼5.74)	0.897	0.039			

OASIS: oxford acute severity of illness score; SOFA: sequential organ failure assessment; APS III: acute physiology score III; BUN: blood urea nitrogen; WBC: white blood cell; RDW: red blood cell distribution width; RA: red blood cell distribution width-albumin ratio; CHF: chronic heart failure; OR: odds ratio.

**Table 3:** Predictive performances and validation of the nomogram.

Predictive model	AUC	95% CI	*P* value	NRI	95% CI	*P* value	IDI	95% CI	*P* value
Training cohort									
Nomogram	0.891	0.846∼0.936	<0.01						
SOFA	0.79	0.716∼0.863	<0.01	0.35	0.119∼0.581	<0.01	0.199	0.101∼0.296	<0.01
OASIS	0.746	0.672∼0.819	<0.01	0.407	0.173∼0.64	<0.01	0.249	0.15∼0.348	<0.01
APS III	0.837	0.777∼0.896	<0.01	0.25	0.008∼0.492	0.043	0.159	0.053∼0.266	<0.01

Validation cohort									
Nomogram	0.898	0.814∼0.982	<0.01						
SOFA	0.828	0.747∼0.91	<0.01	0.473	0.139∼0.807	<0.01	0.355	0.143∼0.567	<0.01
OASIS	0.775	0.646∼0.905	<0.01	0.5148	0.18∼0.85	<0.01	0.382	0.195∼0.57	<0.01
APS III	0.796	0.679∼0.913	<0.01	0.372	0.01∼0.754	0.056	0.37	0.17∼0.572	<0.01

SOFA: sequential organ failure assessment; OASIS: oxford acute severity of illness score; APS III: acute physiology score III; NRI: net reclassification improvement; IDI: integrated discrimination improvement.

## Data Availability

The datasets are publicly available in https://mimic.physionet.org/.
